# An observational, sequential analysis of the relationship between local economic distress and inequities in health outcomes, clinical care, health behaviors, and social determinants of health

**DOI:** 10.1186/s12939-023-01984-6

**Published:** 2023-09-05

**Authors:** William B Weeks, Ji E Chang, José A Pagán, Ann Aerts, James N Weinstein, Juan Lavista Ferres

**Affiliations:** 1 AI for Good Lab, Microsoft, Redmond, WA USA; 2 NYU School of Global Public Health, New York, NY USA; 3 Novartis Foundation, Basel, Switzerland; 4 Microsoft Research, Redmond, WA USA

**Keywords:** Population health, Health equity, Socio-economic status, Social determinants of health

## Abstract

**Background:**

Socioeconomic status has long been associated with population health and health outcomes. While ameliorating social determinants of health may improve health, identifying and targeting areas where feasible interventions are most needed would help improve health equity. We sought to identify inequities in health and social determinants of health (SDOH) associated with local economic distress at the county-level.

**Methods:**

For 3,131 counties in the 50 US states and Washington, DC (wherein approximately 325,711,203 people lived in 2019), we conducted a retrospective analysis of county-level data collected from County Health Rankings in two periods (centering around 2015 and 2019). We used ANOVA to compare thirty-three measures across five health and SDOH domains (Health Outcomes, Clinical Care, Health Behaviors, Physical Environment, and Social and Economic Factors) that were available in both periods, changes in measures between periods, and ratios of measures for the least to most prosperous counties across county-level prosperity quintiles, based on the Economic Innovation Group’s 2015–2019 Distressed Community Index Scores.

**Results:**

With seven exceptions, in both periods, we found a worsening of values with each progression from more to less prosperous counties, with least prosperous counties having the worst values (ANOVA p < 0.001 for all measures). Between 2015 and 2019, all except six measures progressively worsened when comparing higher to lower prosperity quintiles, and gaps between the least and most prosperous counties generally widened.

**Conclusions:**

In the late 2010s, the least prosperous US counties overwhelmingly had worse values in measures of Health Outcomes, Clinical Care, Health Behaviors, the Physical Environment, and Social and Economic Factors than more prosperous counties. Between 2015 and 2019, for most measures, inequities between the least and most prosperous counties widened. Our findings suggest that local economic prosperity may serve as a proxy for health and SDOH status of the community. Policymakers and leaders in public and private sectors might use long-term, targeted economic stimuli in low prosperity counties to generate local, community health benefits for vulnerable populations. Doing so could sustainably improve health; not doing so will continue to generate poor health outcomes and ever-widening economic disparities.

## Contributions to the literature

- Since local economic distress is associated with worse health outcomes, policymakers should consider returns to health as a motivator for improving economic distress.
- The potential magnitude of the impact of reducing economic disparities on clinical quality, outcomes, and health behaviors should be considered when investing to improve local economic conditions.
- Targeted economic stimuli to generate local, community health benefits for vulnerable populations living in the least prosperous areas may be an effective way to improve population health.

## Background

Socioeconomic status has long been associated with population health and health outcomes in industrial countries. [1–3] In the United States (US), among older adults enrolled in traditional Medicare, living in areas of high local economic distress (an index compiled from seven measures of local economic activity obtained from US Census Bureau, US Bureau of Labor Statistics, and American Community Survey data [4] has been associated with higher per-capita Medicare expenditures, lower care quality, higher mortality, [5] and less use of recommended services. [6] Improving local economic conditions in the US is associated with improved health outcomes in Medicare [7] and non-Medicare populations. [8].

The distribution of economic prosperity among US communities has undergone significant changes in recent decades, resulting in heightened inequality in local economic prosperity. [9] This has led to a growing interest in developing policies and resources that support both “places” and “people,“ particularly in underserved communities. [10,11] Such policies recognize that socio-economic conditions are significant determinants of health and that ameliorating social determinants of health (SDOH) - the non-medical factors that influence health outcomes - may improve population health. [12] However, formulating an effective policy response requires identifying and targeting areas where interventions are most greatly needed, are achievable, and might have the largest impact on health equity.

To identify characteristics associated with such areas, we sought to identify cross-sectional and longitudinal inequities in health, clinical care, health behaviors, and SDOH associated with local economic distress at the county level, using 2015 and 2019 data from County Health Rankings.

## Methods

### Data collection and aggregation

For 3,131 counties in the 50 US states and Washington, DC (wherein 325,711,203 people lived in 2019), we obtained Distressed Communities Index (DCI) scores from the Economic Innovation Group. [4] Constructed from seven measures of local economic distress collected from the US Census, US Bureau of Labor Statistics, and the American Community Survey over the period 2015–2019, DCI scores are ranked percentiles that are equally distributed and range from 0 (most prosperous) to 100 (least prosperous). [4] For those counties, we collected 33 county-level attributes obtained from the 2015–2022 County Health Rankings [13] across five health and SDOH domains: Health Outcomes, Clinical Care, Health Behaviors, Physical Environment, and Social and Economic Factors. We limited measures to those available in both (approximately) 2015 and 2019, in essence using a convenience sample of available measures that approximately bookended the time period over which data were used to calculate DCI scores. Table 1 provides the measure name, definition, measure value orientation, periods of data collection, and year interval, across the five domains. Table 2 shows the original sources from which County Health Rankings obtained these measures.

### Analysis

In both years, we compared the health and SDOH measures across prosperity quintiles, defined by county-level DCI scores (there were 626 counties in the most prosperous, highly prosperous, average, and unprosperous quintiles and 627 counties in the least prosperous quintile) using Analysis of Variance (ANOVA). We calculated the ratio of values for the least to the most prosperous county quintiles. Further, for each prosperity quintile, we calculated the change in values for each prosperity quintile between 2015 and 2019. Finally, we calculated the ratio of values for the least to the most prosperous counties between the first and second period and provided an indication of whether the gap between the least and most prosperous counties was widening, narrowing, or staying the same. We used SPSS v 28 (released 2022, Armonk, NY: IBM Corporation) for all analyses.

## Results

In 2019, we found a progressive worsening of values with movement to a less prosperous quintile for all except five measures (ANOVA p < 0.001 for all measures) (Table 3). All Health Outcomes values got progressively worse with worsening county-level prosperity. For example, diabetes is least prevalent in the most prosperous quintile of counties (8.84%); its prevalence progressively increases as prosperity decreases, reaching a peak in the least prosperous quintile of counties (13.49%). All Clinical Care metrics got progressively worse with worsening county-level prosperity, although the mental health workforce measure did not do so in a strictly progressive manner (the second least prosperous quintile had the worst value). All Health Behavior metrics got progressively worse with lowering county-level prosperity except for excessive drinking, which showed the opposite pattern: 20.84% of the adult population reported excessive drinking in the most prosperous quintile of counties, but that proportion progressively fell with worsening prosperity to reach a nadir of 16.43% in the least prosperous quintile of counties. In the Physical Environment domain, measures of air quality and severe housing problems were worst in the least prosperous two quintiles, but there was not a progressive pattern of worsening. All Social and Economic Factors metrics got progressively worse with lowering county-level prosperity except for the membership association rate, where there was an inverse U-shaped pattern, with the least economically prosperous quintile having the worst value.

**Table 1:** Measures collected, with domain, definition, orientation, periods obtained, and year interval between periods

Domain	Measure name	Definition	Higher is…	First period	Second period	Year interval
**Health Outcomes**	Diabetes prevalence	Percentage of adults aged 20 + with diagnosed diabetes	Worse	2015	2019	4
	Fair or poor health	Age-adjusted percentage of adults in fair or poor health	Worse	2015	2019	4
	Frequent mental distress	Percentage of adults reporting 14 + days of poor mental health per month	Worse	2015	2019	4
	Frequent physical distress	Percentage of adults reporting 14 + days of poor physical health per month	Worse	2015	2019	4
	Life expectancy	Life expectancy at birth in years	Better	2015-17	2018-20	3
	Low birth weight	Percentage of live births that are < 2500 g	Worse	2010-16	2014-20	3
	Mentally unhealthy days	Age-adjusted average number of mentally unhealthy days in the last 30 days	Worse	2015	2019	4
	Physically unhealthy days	Age-adjusted average number of physically unhealthy days in the last 30 days	Worse	2015	2019	4
	Premature mortality	Age-adjusted number of deaths among residents under age 75 per 100,000	Worse	2015-17	2018-20	3
	Years potential life lost	Age-adjusted years of potential life lost before age 75 per 100,000 population	Worse	2015	2018-20	4
**Clinical Care**	Dental workforce	Ratio of dentists to the population	Better	2015	2019	4
	Mammography screening rate	Percentage of female Medicare enrollees 65–74 that received annual mammogram screening	Better	2016	2019	3
	Mental health workforce	Ratio of mental health providers to the population	Better	2015	2019	4
	PCP workforce	Ratio of primary care physicians to the population	Better	2015	2019	4
	Preventable hospitalization rate	Preventable hospitalizations per 100,000 Medicare enrollees	Worse	2015	2019	4
	Uninsured	Percentage of population under age 65 that is uninsured	Worse	2015	2019	4
	Vaccinated	Percentage of fee-for-service Medicare enrollees that had an annual flu vaccine	Better	2016	2019	3
**Health Behaviors**	Chlamydia cases	Newly diagnosed chlamydia cases per 100,000 population	Worse	2015	2019	4
	Excessive drinking	Percentage of adults reporting binge or heavy drinking	Worse	2015	2019	4
	Food index	Food environment index (0 to 10 point scale, 0 is worst)	Better	2015	2019	4
	Food insecurity	Percentage of population lacking adequate access to food	Worse	2015	2019	4
	Insufficient sleep	Percentage of adults reporting fewer than 7 h of sleep on average	Worse	2015	2019	4
	Limited healthy food access	Percentage of population who are low-income and do not live close to a grocery store	Worse	2016	2018	2
	Obesity	Percentage of adults aged 20 + with a BMI ≥ 30	Worse	2015	2019	4
	Physical inactivity	Percentage of adults aged 20 + reporting no leisure time physical activity	Worse	2015	2019	4
	Smokers	Percentage of adults who are current smokers	Worse	2015	2019	4
**Physical Environment**	Air quality	Average daily density of fine particulate matter in micrograms per cubic meter	Worse	2014	2018	4
	Severe housing problems	Percentage of households with at least 1 of 4 housing problems	Worse	2012-16	2014-18	5
**Social and Economic Factors**	Child food program participation	Percentage of children enrolled in public schools that are eligible for a free or reduced-price lunch	Worse	2012-16	2016-20	4
	Children in poverty	Percentage of population under age 18 living in poverty	Worse	2015	2019	4
	Deaths due to injury	Number of deaths due to injury per 100,000 population	Worse	2014-15	2018-19	4
	Income inequality	Ratio of household income at the 80th percentile to income at the 20th percentile	Worse	2015	2020	5
	Membership association rate	Number of membership associations per 10,000 population	Better	2011-15	2016-20	5

**Table 2:** Measures collected, with domain and original source of data that was compiled in County Health Reports

Domain	Measure name	Original data source
**Health Outcomes**	Diabetes prevalence	United States Diabetes Surveillance System
	Fair or poor health	Behavioral Risk Factor Surveillance System
	Frequent mental distress	Behavioral Risk Factor Surveillance System
	Frequent physical distress	Behavioral Risk Factor Surveillance System
	Life expectancy	National Center for Health Statistics, Mortality Files
	Low birth weight	National Center for Health Statistics, Natality Files
	Mentally unhealthy days	Behavioral Risk Factor Surveillance System
	Physically unhealthy days	Behavioral Risk Factor Surveillance System
	Premature mortality	National Center for Health Statistics, Mortality Files
	Years potential life lost	National Center for Health Statistics, Mortality Files
**Clinical Care**	Dental workforce	Area Health Resource File
	Mammography screening rate	Mapping Medicare Disparities Tool
	Mental health workforce	Centers for Medicare and Medicaid Services, National Provider Identification
	PCP workforce	Area Health Resource File
	Preventable Hospitalization rate	Mapping Medicare Disparities Tool
	Uninsured	Small Area Health Insurance Estimates
	Vaccinated	Mapping Medicare Disparities Tool
**Health Behaviors**	Chlamydia cases	National center for HIV/AIDS, Viral Hepatitis, STD, and TB prevention
	Excessive drinking	Behavioral Risk Factor Surveillance System
	Food index	USDA Food Environment Atlas
	Food insecurity	Map the Meal Gap
	Insufficient sleep	Behavioral Risk Factor Surveillance System
	Limited healthy food access	USDA Food Environment Atlas
	Obesity	United States Diabetes Surveillance System
	Physical inactivity	United States Diabetes Surveillance System
	Smokers	Behavioral Risk Factor Surveillance System
**Physical Environment**	Air quality	Environmental Public Health Tracking Network
	Severe housing problems	Comprehensive Housing Affordability Strategy Data
**Social and Economic Factors**	Child food program participation	National Center for Education Statistics
	Children in poverty	Small Area Income and Poverty Estimates
	Deaths due to injury	National Center for Health Statistics, Mortality Files
	Income inequality	American Community Survey, 5-year estimates
	Membership association rate	County Business Patterns

**Table 3:** Results for the later collection period (around 2019), by county prosperity quintile. All ANOVA differences across prosperity quintiles p < 0.001. Values in italics did not follow a stepwise worsening of measure value when moving from a higher to a lower prosperity quintile. Values in bold indicate measures where there was improvement in measure values when moving from a higher to a lower prosperity quintile

Domain	Measure	County prosperity quintile				
		Most	High	Average	Low	Least
**Health Outcomes**	Diabetes prevalence	8.84	9.68	10.34	11.57	13.49
	Fair or poor health	15.70	18.07	19.83	22.67	26.79
	Frequent mental distress	13.70	14.84	15.75	17.04	18.50
	Frequent physical distress	11.13	12.43	13.39	14.83	16.87
	Life expectancy	79.82	78.21	77.01	75.65	73.83
	Low birth weight	7.20	7.47	7.85	8.60	9.92
	Mentally unhealthy days	4.34	4.60	4.83	5.17	5.51
	Physically unhealthy days	3.62	3.98	4.26	4.65	5.20
	Premature mortality	309	374	421	479	571
	Years potential life lost	6331	7748	8800	9223	9223
**Clinical Care**	Dental workforce	60.23	51.47	46.02	41.81	35.26
	Mammography screening rate	45.92	44.87	42.75	39.78	36.71
	*Mental health workforce*	*194*	*170*	*154*	*137*	*150*
	PCP workforce	71.97	58.03	53.29	47.96	40.66
	Preventable hospitalization rate	32.88	35.48	38.75	43.77	51.16
	Uninsured	9.03	10.82	11.71	13.46	14.63
	Vaccinated	50.11	45.09	42.45	40.34	36.76
**Health Behaviors**	Chlamydia cases	339	367	378	442	558
	**Excessive drinking**	**20.84**	**20.47**	**19.57**	**18.03**	**16.43**
	Food index	8.45	7.86	7.54	7.01	6.41
	Food insecurity	9.46	11.35	12.74	14.65	17.23
	Insufficient sleep	34.25	35.29	36.41	38.09	40.07
	Limited healthy food access	5.70	7.84	8.33	9.81	10.76
	Obesity	31.89	34.40	35.55	37.22	39.54
	Physical inactivity	24.61	27.88	29.83	32.75	36.70
	Smokers	16.37	18.87	20.30	21.91	24.34
**Physical Environment**	*Air quality*	*7.96*	*7.88*	*7.90*	*8.20*	*8.17*
	*Severe housing problems*	*13.01*	*12.83*	*12.96*	*13.42*	*14.53*
**Social and Economic Factors**	Child food program participation	37.05	46.47	53.01	61.54	73.80
	Children in poverty	10.27	14.59	17.89	21.90	28.71
	Deaths due to injury	74.23	86.10	93.61	98.15	107.64
	Income inequality	4.04	4.25	4.41	4.65	5.20
	*Membership association rate*	*10.42*	*12.29*	*12.72*	*11.65*	*10.36*

Identical patterns were found when examining earlier data (Table 4), with the exception being that the membership association rate was second worst in the least prosperous quintile. When examining changes in measure values between earlier and later data collection periods, most measures demonstrated progressive worsening of values with worsening prosperity, suggesting that inequities increased over time (Table 5). There were several exceptions to this general rule: years potential life lost increased more in higher prosperity quintiles; the preventable hospitalization rate fell as prosperity worsened; the least prosperous quintile experienced the greatest absolute decline in the uninsurance rate; and there was a stepwise reduction in childhood poverty as prosperity decreased. There was no clear pattern in food insecurity, limited healthy food access, air quality, severe housing problems, or the membership association rate. While income equality worsened most in the least prosperous quintile counties, there was not a progressive, stepwise pattern.

When comparing ratios of values in the least to the most prosperous counties in 2015 and 2019, 20 measures demonstrated a widening of the gap between the least and most prosperous counties, 10 demonstrated a narrowing, and 3 remained the same (Table 6).

**Table 4:** Results for the earlier data collection period (around 2015), by county prosperity quintile. All ANOVA differences across prosperity quintiles p < 0.001. Values in italics did not follow a stepwise worsening of measure value when moving from a higher to a lower prosperity quintile. Values in bold indicate measures where there was improvement in measure values when moving from a higher to a lower prosperity quintile

Domain	Measure	County prosperity quintile				
		Most	High	Average	Low	Least
**Health Outcomes**	Diabetes prevalence	9.72	10.76	11.50	12.51	13.65
	Fair or poor health	12.90	14.68	16.20	18.74	22.55
	Frequent mental distress	10.21	10.83	11.41	12.35	13.54
	Frequent physical distress	9.77	10.70	11.46	12.68	14.48
	Life expectancy	80.08	78.64	77.52	76.29	74.74
	Low birth weight	7.15	7.32	7.71	8.53	9.84
	Mentally unhealthy days	3.39	3.55	3.72	3.98	4.26
	Physically unhealthy days	3.29	3.58	3.82	4.19	4.69
	Premature mortality	300	360	400	450	523
	Years potential life lost	5931	7153	7987	9066	9223
**Clinical Care**	Dental workforce	56.26	47.50	42.13	38.45	32.32
	Mammography screening rate	43.75	42.56	40.46	38.16	34.97
	*Mental health workforce*	*148*	*132*	*121*	*103*	*106*
	PCP workforce	71.38	58.49	53.74	48.22	42.15
	Preventable hospitalization rate	44.96	52.67	58.28	65.41	77.74
	Uninsured	9.15	10.84	11.82	13.39	14.90
	Vaccinated	46.89	42.29	40.02	38.30	34.98
**Health Behaviors**	Chlamydia cases	298	328	334	376	477
	**Excessive drinking**	**18.80**	**17.82**	**16.83**	**15.46**	**14.09**
	Food index	8.24	7.76	7.51	7.11	6.49
	Food insecurity	11.20	12.52	13.55	15.22	18.13
	Insufficient sleep	31.23	31.58	32.42	34.01	35.98
	Limited healthy food access	5.50	8.12	8.73	9.70	10.71
	Obesity	28.91	31.43	32.33	33.34	34.38
	Physical inactivity	21.14	24.23	25.94	27.86	29.36
	Smokers	15.08	16.59	17.58	19.01	21.17
**Physical Environment**	*Air quality*	*8.99*	*8.76*	*8.85*	*9.26*	*9.27*
	*Severe housing problems*	*13.59*	*13.39*	*13.43*	*13.83*	*14.97*
**Social and Economic Factors**	Child food program participation	37.74	47.23	53.22	61.09	70.30
	Children in poverty	13.77	18.77	22.34	26.97	34.38
	Deaths due to injury	65.53	78.03	84.29	87.47	96.80
	Income inequality	4.10	4.32	4.45	4.65	5.10
	*Membership association rate*	*11.70*	*14.76*	*15.58*	*14.28*	*12.74*

**Table 5:** Change in measure values between the earlier and later data collection period, by county prosperity quintile. Values in italics did not follow a stepwise worsening of measure value when moving from a higher to a lower prosperity quintile. Values in bold indicate measures where there was improvement in measure values among the least prosperous counties

Domain	Measure	County prosperity quintile				
		Most	High	Average	Low	Least
**Health Outcomes**	Diabetes prevalence	-0.88	-1.08	-1.16	-0.94	-0.16
	Fair or poor health	2.80	3.38	3.63	3.93	4.24
	Frequent mental distress	3.49	4.00	4.34	4.69	4.96
	Frequent physical distress	1.36	1.73	1.93	2.15	2.39
	Life expectancy	-0.26	-0.43	-0.52	-0.64	-0.91
	Low birth weight	0.05	0.15	0.15	0.06	0.08
	Mentally unhealthy days	0.95	1.05	1.12	1.19	1.24
	Physically unhealthy days	0.33	0.40	0.44	0.46	0.51
	Premature mortality	9.08	14.17	21.68	28.60	47.73
	***Years potential life lost***	***400***	***595***	***812***	***157***	***0***
**Clinical Care**	Dental workforce	3.97	3.96	3.90	3.36	2.95
	*Mammography screening rate*	*2.17*	*2.31*	*2.29*	*1.62*	*1.74*
	*Mental health workforce*	*45.89*	*38.43*	*32.95*	*33.53*	*43.41*
	*PCP workforce*	*0.58*	*-0.46*	*-0.45*	*-0.26*	*-1.49*
	**Preventable hospitalization rate**	**-12.08**	**-17.19**	**-19.53**	**-21.64**	**-26.57**
	**Uninsured**	**-0.13**	**-0.02**	**-0.11**	**0.07**	**-0.26**
	Vaccinated	3.22	2.80	2.43	2.04	1.78
**Health Behaviors**	Chlamydia cases	41.05	39.02	43.71	65.99	81.65
	*Excessive drinking*	*2.04*	*2.66*	*2.74*	*2.57*	*2.34*
	Food index	0.21	0.11	0.03	-0.10	-0.08
	*Food insecurity*	*-1.75*	*-1.17*	*-0.82*	*-0.57*	*-0.90*
	Insufficient sleep	3.02	3.71	3.99	4.08	4.08
	*Limited healthy food access*	*0.20*	*-0.28*	*-0.40*	*0.11*	*0.05*
	Obesity	2.99	2.97	3.22	3.88	5.15
	Physical inactivity	3.47	3.65	3.90	4.89	7.34
	Smokers	1.29	2.27	2.72	2.90	3.17
**Physical Environment**	*Air quality*	*-1.04*	*-0.88*	*-0.95*	*-1.06*	*-1.10*
	*Severe housing problems*	*-0.57*	*-0.56*	*-0.46*	*-0.41*	*-0.44*
**Social and Economic Factors**	Child food program participation	-0.68	-0.76	-0.22	0.44	3.49
	**Children in poverty**	**-3.51**	**-4.18**	**-4.45**	**-5.08**	**-5.66**
	Deaths due to injury	8.70	8.08	9.31	10.68	10.84
	*Income inequality*	*-0.06*	*-0.07*	*-0.04*	*0.00*	*0.10*
	*Membership association rate*	*-1.28*	*-2.47*	*-2.86*	*-2.63*	*-2.38*

**Table 6:** Ratios of values in the least to the most prosperous counties in 2015 and 2019 and an indication of whether the gap between least and most prosperous counties is widening, narrowing, or staying the same

Domain	Measure	Higher is.	Ratio of least to most prosperous county values		Between 2015 and 2019, gap between least and most prosperous counties is…
			2015	2019	
**Health Outcomes**	Diabetes prevalence	Worse	1.40	1.53	Widening
	Fair or poor health	Worse	1.75	1.71	Narrowing
	Frequent mental distress	Worse	1.33	1.35	Widening
	Frequent physical distress	Worse	1.48	1.52	Widening
	Life expectancy	Better	0.93	0.92	Widening
	Low birth weight	Worse	1.38	1.38	Unchanged
	Mentally unhealthy days	Worse	1.26	1.27	Widening
	Physically unhealthy days	Worse	1.42	1.44	Widening
	Premature mortality	Worse	1.75	1.85	Widening
	Years potential life lost	Worse	1.56	1.46	Narrowing
**Clinical Care**	Dental workforce	Better	0.57	0.59	Narrowing
	Mammography screening rate	Better	0.80	0.80	Unchanged
	Mental health workforce	Better	0.72	0.77	Narrowing
	PCP workforce	Better	0.59	0.56	Widening
	Preventable hospitalization rate	Worse	1.73	1.56	Narrowing
	Uninsured	Worse	1.63	1.62	Narrowing
	Vaccinated	Better	0.75	0.73	Widening
**Health Behaviors**	Chlamydia cases	Worse	1.60	1.65	Widening
	Excessive drinking	Worse	0.75	0.79	Widening
	Food index	Better	0.79	0.76	Narrowing
	Food insecurity	Worse	1.62	1.82	Widening
	Insufficient sleep	Worse	1.15	1.17	Widening
	Limited healthy food access	Worse	1.95	1.89	Narrowing
	Obesity	Worse	1.19	1.24	Widening
	Physical inactivity	Worse	1.39	1.49	Widening
	Smokers	Worse	1.40	1.49	Widening
**Physical Environment**	Air quality	Worse	1.03	1.03	Unchanged
	Severe housing problems	Worse	1.10	1.12	Widening
**Social and Economic Factors**	Child food program participation	Worse	1.86	1.99	Widening
	Children in poverty	Worse	2.50	2.80	Widening
	Deaths due to injury	Worse	1.48	1.45	Narrowing
	Income inequality	Worse	1.24	1.29	Widening
	Membership association rate	Better	1.09	0.99	Narrowing

## Discussion

In the late 2010s in the US, less prosperous counties had worse values than more prosperous ones in 29 of 33 measures of Health Outcomes, Clinical Care, Health Behaviors, the Physical Environment, and Social and Economic Factors; for 26 of those measures, during a time of economic growth across the US, there was a progressive worsening of measure values with each move from a higher to a lower prosperity county. Further, with four exceptions, measures in the least prosperous counties worsened more than those in the most prosperous counties between approximately 2015 and 2019, suggesting that inequities in health and SDOH measures associated with economic prosperity increased during that period.

The general stepwise nature of the relationship between increasing economic distress and the measures we studied suggests a structural relationship that has led to a systemic and sequential worsening of health as one descends the economic prosperity ladder. Our findings support that local economic prosperity is associated with health status, health outcomes, and health care quality in Medicare fee-for-service patients [5,6] and other populations [3, 14–18]. Further, for most of the measures we examined, the gap between the least and most prosperous counties widened in the immediate pre-pandemic period.

Not all measures demonstrated a stepwise worsening with increasing local economic distress. Physical Environment and Social and Economic Factors measures showed distinct patterns, both cross-sectionally and over time. Nonetheless, measures in the Physical Environment were invariably worse in the least prosperous counties.

It is worth noting that we found an inverse relationship between reporting of excessive drinking and local economic prosperity, though binge drinking increased across all prosperity quintiles between 2015 and 2019. Indeed, binge drinking is more common in members of higher household incomes and those with greater educational attainment. [19] It is possible that binge drinking is more culturally accepted in higher-income groups, or that alcohol consumption is relatively expensive compared to other drugs. The inverse relationship between price increases and alcohol use has long been documented; [20] studies of the relative prices of alcohol and illicit drugs, particularly in lower prosperity areas, should be conducted.

Our study has several limitations. First, our results are derived from data in two relatively close time periods in a relatively stable financial time; studies of different time periods may have different results. Importantly, we evaluated periods before the COVID-19 pandemic and reports suggest that economic and health inequities have increased since COVID-19 began; [21] therefore, our results might underestimate current inequities. Further, analyses of other time periods – for instance, during the 2008 financial crisis – might generate different results. Second, measures are not adjusted for local demographic factors that may impact measure values. For example, Blacks are more likely than Whites to have diabetes, [22] lower life expectancy, [23] and low birth weight babies; [24] Blacks are also more likely than Whites to live in areas with lower economic prosperity and may experience different outcomes than Whites living in the same economic conditions after admission for heart failure. [25] While demographic factors may partially explain our findings (for instance, among 25–34 year old participants in the Behavioral Risk Factor Surveillance System between 2009 and 2012, after demographic adjustments county-level economic opportunity was found to independently contribute to measures of Health Outcomes and Health Behaviors [26], demographic adjustment offers policymakers few pragmatic solutions if health equity is to be color-blind: changing the demographic makeup of a county cannot be a reasonable policy platform. While demographic adjustment is important in real-world policy development, in this observational study, we did not make demographic adjustments because we were concerned that demographic adjustment might inadvertently justify a demographic group’s obtaining lower quality care or less care access. Third, we limited our evaluation to county-level quintiles of economic prosperity and did not evaluate other potentially contributing factors, such as rural-urban disparities or geographic variation in health outcomes. To be sure, it is likely that more rural counties and more counties in the southeastern United States more persistently and commonly experience local economic distress. [27] Nonetheless, that reality does not refute our findings: it suggests that more rural and southeastern counties experience worse measures of health outcomes, clinical care measures, health behaviors, the physical environment, and social and economic factors. Fourth, our analysis was performed at the county quintile level: we did not seek to identify outliers, such as low prosperity counties with excellent health outcomes or vice-versa. In future work, particularly should robust longitudinal data become available, such analyses might give insights into reasons why counties become more prosperous or healthier and might identify causal pathways between population health and local prosperity. Finally, we did not have access to data that might have explored the relationship between our findings and the degree to which: particular measures – for instance, life expectancy or premature mortality – might be amenable to intervention by targeted risk factor modification at the population level; [28] the local political environment or other unmeasured factors might contribute to our findings; or the influence of geographically proximal economic distress might influence local economic distress. Each of these areas warrants further research that likely would require multi-decade datasets, across a variety of global economic conditions.

Despite these limitations, our findings suggest that investment in low prosperity qualified ‘economic opportunity zones’ might not only improve local economic conditions, but also improve community health, [29] thereby reducing health inequities, regardless of the demographic makeup of those areas. While our findings are associative and not causative, aforementioned studies used natural experimental methods and suggest that improving economic conditions might generate health benefits, rather rapidly. [7,8] Should more longitudinal and robust data become available, policymakers might be able to model the impact that targeted efforts to improve local economic conditions might have on measures of local population health.

## Conclusions

Our findings suggest that local economic prosperity may serve as a proxy for the health and SDOH status of the community. Communities operate within the context of federal and state policies that shape local economic conditions including the allocation of resources and strategic priorities. [9] Together, policymakers, health plans, health systems, public health leaders, and leaders in corporate America should consider long-term, targeted economic stimuli to generate local, community health benefits for vulnerable populations living in the least prosperous areas.

## Data Availability

Data used in the study are publicly available at https://eig.org/distressed-communities/. The EIG data – which aggregate data from the American Community Survey, the US Bureau of Labor, and the US Census, and does not include individual-level data - can be purchased for use by researchers or policymakers. All methods were carried out in accordance with relevant guidelines and regulations. Because there are no individual data elements and the data are sourced from publicly available data, the study is not considered Human Subjects research and therefore does not require IRB approval. Similarly, because data are publicly available and are not individual-level, no informed consent was required. Microsoft paid EIG $2000 (the cost for any business to purchase these data) to be able to use these data for this study. And https://www.countyhealthrankings.org/explore-health-rankings/county-health-rankings-measures.

## Abbreviations

US: United States
SDOH: Social determinants of health
DCI: Distressed Communities Index
ANOVA: Analysis of variance
